# An Empirical Analysis of Audio-Visual Teaching and Network Multi-Modal Learning Environment Theory for English Majors

This article has been retracted.

**DOI:** 10.1155/2022/5000501

**Published:** 2022-08-11

**Authors:** Yuanyuan Gao

**Affiliations:** English Department, Changzhi University, Changzhi, Shanxi 046011, China

## Abstract

In order to further investigate the network multi-modal learning environment to promote students' ability to English audio-visual effects and improve the quality of teaching effect, an empirical analysis of audio-visual teaching and network multi-modal learning environment theory for English majors was proposed in the research. The 98 students were chosen as the experiment objects from two classes in the same school. They were divided into the experiment class and the control class. The students in the experiment class were taught according to the teaching model based on network multi-modal learning environment theory. SPSS19.0 software was used to analyze the scores before and after the experiment. After 3 months of experiment teaching, the average score of the post-test of the experiment class was 13.65 points, 2.23 points higher than 11.42 points before the test. The average score of the control class was 11.08 points, 0.1 points lower than 11.18 points before the test. It could be seen that the teaching method based on a network multi-modal learning environment was more conducive to improving the audio-visual performance and the teaching effectiveness of English majors.

## 1. Introduction

In recent years, with the continuous development of science and technology, especially in the field of education and the development of high-tech media information technology, multimedia technology has been widely used in classroom teaching and textbook compilation has begun to present a multi-modal development mode [1]. In the network environment background, the teachers in the teaching process can choose more and more teaching methods and means. The fusion of multi-modal learning environment theory and contemporary classroom teaching can better reflect the advantages. In the teaching process, teachers can use multi-modal learning theory more flexibly and accurately to mobilize students' various senses. And boring knowledge or text content is transformed into more attractive image text or video content. Such teaching media resources, which combine pictures, sounds and videos, are more conducive to improving students' interest in learning, as well as their subconscious learning intensity, so that students can have a deeper understanding of knowledge [2]. The focus of the research is to explore how to improve the audio-visual teaching quality and learning effectiveness of English majors with the help of network multi-modal learning theory through empirical research.

## 2. Literature Review

The multi-modal teaching theory combined with the traditional listening teaching was investigated. They believed that the interaction between the different models and the effect of the different modal interactions in the process of listening teaching also produced a different effect. Students' listening comprehension ability in the application of multi-modal teaching mode could be improved more significantly. How to provide a multi-modal interactive learning environment including text, voice, and video for second language learners was discussed. And the fact that students were more interested in listening and easier to understand the multimedia listening materials with subtitles was verified. The teaching methods aiming at helping students improve their listening comprehension ability and learn vocabulary in the multimedia context were summarized [3]. Assistance was any form, such as visual, auditory and textual materials, which could be presented synchronously or asynchronously on a computer screen to aid language teaching. It was found that both synchronous and asynchronous text visual and auditory computer-aided learning were more conducive to improving students' listening comprehension.

Foreign scholars initially investigated the promotion of second language subtitles to students' listening development. In recent years, they investigated the improvement of listening comprehension ability in a multimedia context. With the development of multimedia technology, it provided the prerequisite for the emergence of various teaching modes [4].

In the early years, a group of scholars tried to use multimedia technology and video materials in listening teaching (Figure 1). For example, it was believed that playing video materials in the process of listening teaching could improve students' listening levels. The wide application of multimedia and the feasibility of classroom teaching by using film and other film materials and the necessity for teachers to reform the traditional listening class were discussed. The students' listening motivation and the changes in their listening level by using English movies as materials in visual English class were also explored [5]. The experiment results showed that the experiment students' enthusiasm for English listening learning had been improved and the students' agility of thinking had been stimulated. Some scholars used the multi-modal teaching method in the teaching of business English majors in higher vocational colleges and the effect was very good. With the help of the multi-modal teaching mode reform of the college audio-visual speaking curriculum, it was found that students' comprehensive application ability of English was improved effectively. Listening and speaking ability also improved significantly in the process, and the initiative of English learning showed a rising trend [6]. It showed that the multi-modal audio-visual teaching mode played an important role in the reform process. An empirical investigation on listening teaching in a multimedia environment was made, which pointed out that when visual information and auditory information corresponded to each other in the listening process, it played a positive role in improving the listening comprehension ability. They tried to make different modes cooperate in listening training and found that it was of great help to improve the listening level of English majors. Moreover, they found that the multi-modal teaching mode could also improve learners' multi-literacy ability [7].

Learning from the research results of foreign scholars, according to the actual situation of China's current education and teaching, domestic scholars introduced a multi-modal into China's foreign language teaching research to promote its development. However, there are few listening teaching research involving business English majors in vocational colleges. At the same time, the rapid development of modern multimedia network technology in China also provides guaranteed conditions for the development of multi-modal teaching, which makes the effect of multi-modal teaching more obvious [8].

## 3. Experiment Design of Audio-Visual Teaching Based on Network Multi-Modal Learning Environment Theory

### 3.1. Research Objects and Methods

In the research, two classes were selected from a middle school to form the Experiment Class and the Control Class. One class was designated as the Experiment Class with 48 students and the other class as the Control Class with 50 students. In order to ensure the validity of the experiment results, the teaching accuracy of the audio-visual speaking course in the two classes was kept the same [9].

Through the pretest, it was confirmed that the two classes were parallel classes. One class was randomly selected as the Experiment Class and the other as the Control Class. Before and after the listening test, the listening scores of the two classes were counted. And the independent sample *T* test was conducted with SPSS 19.0 software to sort out and analyze the comparison and changes of the listening scores of the students in the two classes [10].

Before and after the experiment, the learning motivation situation of the Experiment Class students in the current listening class and whether the listening learning motivation of the Experiment Class students changed after a period of multi-modal listening teaching were investigated by questionnaire. The interview survey mainly focused on the change in students' motivation for multi-modal listening teaching and the teaching suggestions for the future of multi-modal listening teaching [11].

In order to test the influence of multi-modal listening teaching mode on the change of students' listening learning motivation, based on the specific situation of students' listening learning, the questionnaire was made and revised. The revised questionnaire was divided into seven dimensions with 27 questions in total. SPSS 19.0 software was used to measure the reliability of the questionnaire. As can be seen from Table 1, the Alpha coefficient of the questionnaire survey is 0.958 > 0.7, indicating that the data of the questionnaire scale has high consistency. That is, the data has high credibility [12].

In Table 2, the KMO value is 0.729, which is more than 0.7, indicating that the sample size meets the requirements and the data is suitable for factor analysis. *P* value of Bartlett's sphericity test in the table is 0.000, less than 0.01. The above data indicate that the scale has a good validity [13].

### 3.2. Empirical Research Process

The experiment lasted for 3 months and the listening part of six modules in Module3-Module8 of the second volume of Grade 9 of the Foreign Research Edition was taken as the teaching content. For each module of the listening class, a multi-modal method will be adopted for listening teaching in the Experiment Class, while the traditional listening teaching method will still be adopted in the Control Class. The experiment process included the experiment preparation stage, experiment implementation stage, and post-experiment stage, and the specific process was as follows [14].

#### 3.2.1. Design of Multi-Modal Listening Teaching Mode for the Experiment Class

In the pre-listening stage, multi-modal means such as theme-related video clips, music, multi-modal courseware, and props were used to stimulate students' multi-senses, arouse their listening interest, and guide students to actively participate in classroom activities. The prelistening prediction was guided by multi-modal means to pave the way for background knowledge and clear the hearing barrier [15]. Teachers create visual stimulation and auditory stimulus mainly by showing more modal courseware, supplemented by rich body movements or the physical display. Teachers guided the students to carry on predictions related to the topic content before the listening and helped the students activate existing knowledge, which could sweep hearing impairment. At the beginning of the class, the teacher played a funny video about Mr. Bean helping patients with heart attacks. The students laughed many times during the five minutes of the video. After the video was played, the teacher controlled the classroom atmosphere and led the students to say the theme of the listening lesson: Accident and First Aid. By using visual and auditory modes, the teacher played the content that the students were familiar with to arouse the students' interest in listening.

After listening, the teacher showed the pictures from the textbook on the screen and gave Table 3 to ask the students to work in groups. In the group, students made reasonable associations by observing pictures and combining them with charts. After completing the table, they discussed and described an accident report together. And students were invited to present on the stage [16].

#### 3.2.2. Traditional Listening Teaching Design of the Control Class

Before listening, the teacher introduced the listening topic and related knowledge to the students by asking questions or other ways. The teacher presented the new words and read them. Listening: The teacher played the listen and the students listened. The teacher judged the playing times according to students' reactions. Students completed the questions as they listened. Post-listening: The teacher organized students to check the answers, emphasized the knowledge points in the material, and asked students to master new knowledge through reading the listening materials together [17].

## 4. Experiment Analysis and Discussion of Results

### 4.1. Questionnaire Data Collation and Analysis of Students' Listening Motivation

#### 4.1.1. Collation and Analysis of Questionnaire Survey Results before the Experiment

The 27 questions in the questionnaire before the experiment were investigated from five dimensions (intrinsic interest, scores, learning situation, going abroad, and personal development). A total of 48 questionnaires were sent out and 48 were recovered, and all of them were valid. Specific data analysis is shown in Table 4:

As can be seen from Table 4, in terms of internal interest, a large number of students chose the two options of “Not sure” and “Relatively disagree,” indicating that most of them were not sure whether they were interested in English listening learning, or the current listening class could not arouse students' interest in learning [18].

As can be seen from Table 5, 10.42% of the students thought their listening scores were good and they were confident to face the upcoming high school entrance examination. 12.5% of the students could be engaged in the listening class and concentrate on the listening class. 8.33% of the students had great learning motivation and high listening scores in the current listening classes. 12.5% of the students thought they could successfully pass all kinds of English exams in the future [19].

As can be seen from Table 6, 18.75% of the students believed that teachers designed rich classroom activities for students in listening class and encouraged students to spread their thinking through cooperation. 6.3% of the students thought that in their listening classes, teachers paid more attention to the development of students' ability by combining listening teaching with students' real life. Thus, in the current English listening class, teachers rarely consider the creation of problem situations for students and do not pay attention to the divergence between students' thinking and students' ability to solve problems [20]. In this way, it is difficult to stimulate students' participation in class and students accept knowledge passively, which is not good.

As can be seen from Table 7, 8.3% of the students were confident of passing the future overseas examination with excellent results. 10.42% of the students believed that they had learned a lot about travel in listening classes, so they believed that they could communicate normally when traveling abroad [21]. 10.42% of the students were confident about taking TOEFL in the future. 10.42% of the students thought that their listening score was good and they would like to emigrate abroad in the future. 14.58% of the students believed that they had learned a lot of oral expressions in the listening class and could communicate with foreigners normally. It can be seen that more than 80% of the students chose “Not sure” and “Relatively disagree” in terms of “Going abroad.” Students held uncertain or negative views that listening teaching could help them to study abroad, travel and employment in the future. And in this question, there were relatively more students who chose the option of “Not sure.”

As can be seen from Table 8, 25% of the students agreed that the current listening courses could help them get good scores in future job-hunting exams. 10.42% of the students believed that their listening performance was good and listening classes at present could help them find a good job in the future. 4.17% of the students could understand English articles and dialogues, and believed that they would have more advantages in going abroad or job-hunting in the future. 4.17% of the students believed that they could express their own opinions or understand others well in daily oral communication. It could be seen that in terms of “Personal development,” more than 80% of the students believed that the current listening courses did not promote students' personal development in the future and the current listening courses did not help students' future development.

#### 4.1.2. Collation and Analysis of Questionnaire Survey Results after the Experiment

After 3 months of multi-modal listening teaching, the same questions as the questionnaire before the experiment were used to investigate students' learning motivation for multi-modal English listening teaching from five dimensions (intrinsic interest, scores, learning situation, going abroad, and personal development). A total of 48 questionnaires were sent out and 48 were recovered. All of them were valid.

It can be seen from Table 9 that after 3 months of multi-modal listening teaching, 68.75% of the students were willing to take the initiative to practice listening. 70.84% of the students said they could understand more listening content and 62.5% said they were willing to complete English listening exercises prescribed by the school. 56.3% of the students said they would like to know more about the English-speaking people and their culture and they like listening more and more. 70.83% of the students expressed that the multi-modal listening class was very interesting and they were more interested in English learning. 72.92% of the students said they like English and the multi-modal listening teaching was very interesting. 72.92% of the students said that three months of multi-modal listening teaching could help students get a sense of achievement and the students were more interested in English listening learning. This fully showed that the dimension “Intrinsic interest” from the motivation, more than 70% of students chose “Absolutely agree” and “Relatively disagree” as two options. Thus, most of the students believed that multi-modal listening classroom listening teaching could attract students' attention and could help students to stimulate interest in learning hearing, so as to enhance students' English listening learning motivation.

As can be seen from Table 10 above, 77.08% of the students were confident that they could achieve better results in the upcoming high school entrance examination after three months of multi-modal listening teaching. 85.42% of the students believed that they could concentrate on learning in listening class. 70.83% of the students showed great enthusiasm for learning English and their listening scores were improving. 81.25% of the students believed that they had the confidence to pass the future exams and graduate successfully. This fully showed that from the motivation of the “Scores” dimension, more than 70% of students chose “Absolutely agree” and “Relatively agree” as two options. Most of the students believed that the teaching method of multi-modal listening teaching could help students improve their listening scores and further enhance their motivation for English listening learning.

As can be seen from Table 11, after 3 months of multi-modal listening teaching, 81.25% of the students believed that teachers designed rich classroom activities for students in the listening class and encouraged students to spread their thinking through cooperation. 58.33% of the students believed that the combination of listening teaching and students' real life was considered in their multi-modal listening class. From the perspective of the motivation of learning situation, the multi-modal English listening class took into account the creation of problem situations for students and focused on the cultivation of students' divergent thinking, problem-solving ability, the increase of students' interest in learning, and the improvement of listening learning motivation.

As can be seen from Table 12, 77.08% of the students were confident of getting good scores in the coming overseas examination after three months of multi-modal listening teaching. 75% of the students expressed that after 3 months of multi-modal English listening teaching, they were confident that they could understand English and American languages when traveling abroad. 70.83% of the students said they were more confident to take TOEFL to study abroad. 41.67% of the students said that the multi-modal listening teaching could help students understand more English dialogues and articles and help students realize their dream of emigration or settling down abroad. 37.5% of the students were not sure whether they would emigrate in the future. 77.09% of the students said that they had learned a lot of oral expressions in the multi-modal listening class and were confident in normal communication with foreigners.

As can be seen from Table 13, after three months of multi-modal listening teaching, 87.5% of the students believed that multi-modal listening teaching could help students achieve good scores in the future job examination. 81.25% of the students believed that their listening performance was improving and multi-modal listening classes could help students find a good job in the future. 79.17% of the students believed that they could understand more articles and dialogues in class and believed that they would have more advantages in going abroad or job-hunting in the future. 80.72% of the students believed that multi-modal listening teaching could help students to express their own views or understand others' ideas in daily oral communication, which would be of great help to students' future development. It fully showed that from the dimension of “Personal development” in motivation, multi-modal listening teaching could give students more confidence. And a large number of students believed that they could have better development and be more competitive in the future. They liked this kind of teaching method, which could enhance students' motivation for English listening learning.

### 4.2. Test Data Collection and Analysis of Students' Listening Performance

#### 4.2.1. Comparison of Pretest Listening Scores between the Experiment Class and the Control Class

In order to compare whether there is a significant difference in pretest scores between the Experiment Class and the Control Class, an independent sample *T* test is conducted in the research. And the results are shown in Table 14 and Table 15.

The descriptive statistics of the pretest results of the Experiment Class and the Control Class was shown in Table 14. It can be seen that the average listening score of the Experiment Class was 11.42 and that of the Control Class was 11.18. It can be seen from the value that there was a slight difference between them. The results were shown in Table 15. An independent sample test was carried out on the pretest scores of the Experiment Class and the Control Class. In Levene's test of the variance equation, *P* value was 0.901, higher than 0.05, indicating that the data of the two groups met the homogeneity of variance condition of the independent sample *T* test. Then *t*-test of the mean equation showed that the *P* value was 0.682, higher than 0.05. The above data showed that there was no significant difference in the listening scores of the two classes in the pretest. In other words, the English listening levels of the two classes in the pretest were similar, so the two classes could be determined as parallel classes.

#### 4.2.2. Comparison of Post-test Listening Scores between the Experiment Class and the Control Class

After 3 months of teaching experiments, post-experiment tests were conducted on the students of the Experiment Class and the Control Class, respectively. The post-test scores of the two classes were inputted into SPSS19.0 and the following results were obtained, as shown in Table 16 below.

The descriptive statistics of the post-test results of the Experiment Class and the Control Class was shown in Table 16. It can be seen that the average listening score of the Experiment Class was 13.64 and that of the Control Class was 11.17. In the 3 months of multi-modal after listening teaching mode, students in learning listening had a bigger improvement. However, whether it reached the level of statistical difference is shown in Figure 2.

In Figure 2, the data of the post-test independent sample *t*-test of the Experiment Class and the Control Class showed that the *P* value of the results of the two classes in the post-test by Levene's test of the variance equation was 0.216, higher than 0.05, indicating that the listening scores of the two classes in the post-test met the homogeneity of variance of the independent sample *T* test. The results of the mean equation *T* test showed that the *P* value was 0.000, less than 0.05. The above data showed that there was a significant difference between the listening performance of the Experiment Class and the Control Class. In other words, after 3 months of multi-modal listening teaching, the listening performance of the students in the Experiment Class was significantly higher than that of the students in the Control Class.

## 5. Conclusion

The significance of multi-modal discourse analysis is that it can integrate language and other related resources together. While language expresses and transmits meaning, images, music, colors, and other resource symbols also play an important role in the process of conveying meaning. So humans can generate and express meaning more accurately by using the multi-modal method. Modern communication is no longer a single mode of communication and multi-modal communication has become the mainstream.

Through the collation and analysis of the two questionnaires, it was found that the data of the two questionnaires were different obviously. The post-test questionnaire from seven dimensions strongly proved that the multi-modal listening teaching mode had a significant positive effect on students' listening motivation and the students' listening learning motivation had a significant change. Through the comparison of the test scores, independent sample *T*-value test, and the data of the questionnaire survey between the Experiment Class and the Control Class, it could be concluded that the test listening scores of the Experiment Class were significantly improved after the application of the multi-modal listening teaching mode. The Control Class adopted the traditional listening teaching mode and the test scores did not change significantly. Through the independent sample test, the *P* value of the two classes was less than 0.05, indicating that there was a significant difference between the two classes. The multi-modal listening teaching model can indeed improve the English listening performance of junior high school students. In interviews, through the conversation with my teachers and classmates, the fact that two classes are traditional listening teaching modes before the experiment was made clear. After the teacher and students agreed with the multi-modal theory, it was determined to apply multi-modal means to listening teaching. The multi-modal listening teaching was carried out according to the teachers' suggestions and the actual situation. In the post-test interview, students liked the multi-modal listening teaching mode very much and were more interested and confident to participate in the listening class. The post-test results of the interview assisted to prove the results of the post-test questionnaire. Students also gave some feedback on the multi-modal listening teaching in this stage. Comprehensive data and analysis can be concluded that the multi-modal listening teaching model can enhance students' listening learning motivation and improve junior high school students' listening performance. Moreover, students hold a positive attitude toward the model.

## Figures and Tables

**Figure 1:** Multimedia-assisted English teaching.

**Figure 2:** Independent sample test of the experiment class and the control class.

**Table 1:** Reliability test of questionnaire.

Scale	Dimension	Question items	Cronbach's alpha coefficient	
Scale dimension	Intrinsic interest	7	0.866	0.958
	Scores	2	0.813	
	Learning situation	2	0.752	
	Going abroad	6	0.825	
	Social responsibility	3	0.732	
	Personal development	1	0.775	
	Information media	2	0.761	

**Table 2:** Validity analysis results of questionnaire.

Kaiser–Meyer–Oolkin	729	
Bartlett's sphericity test	The approximate chi-square	1182.629
	Df	352
	Sig	0.000

**Table 3:** Report content.

Accident report
Where
Who
What happened
How the person was hurt

**Table 4:** Statistical situation of “Intrinsic interest” in motivation before experiment.

Question items	Absolutely agree (%)	Relatively agree (%)	Not sure (%)	Relatively disagree (%)	Absolutely disagree (%)
Q1	2.07	22.82	43.71	21.92	8.33
Q3	2.07	8.43	27.01	41.17	20.13
Q4	0.00	37.70	31.15	25.10	6.25
Q5	0.00	10.42	50.00	37.10	2.08
Q6	8.43	11.10	42.17	26.18	10.12
Q14	0.00	6.15	52.01	33.13	8.33
Q19	6.35	10.12	37.51	34.41	10.42

**Table 5:** Statistical situation of “Scores” in motivation before the experiment.

Question items	Absolutely agree (%)	Relatively agree (%)	Not sure (%)	Relatively disagree (%)	Absolutely disagree (%)
Q10	4.77	6.25	25.0	55.18	10.4
Q25	6.75	6.75	16.7	35.5	35.33
Q26	2.78	6.75	14.55	35.58	37.5
Q27	0.00	12.75	22.92	45.92	15.67

**Table 6:** Statistical situation of “Learning situation” in motivation before experiment.

Question items	Absolutely agree (%)	Relatively agree (%)	Not sure (%)	Relatively disagree (%)	Absolutely disagree (%)
Q7	8.53	10.52	43.55	37.55	2.58
Q8	0.00	6.3	14.55	33.53	45.53

**Table 7:** Statistical situation of motivation “Going abroad” before the experiment.

Question items	Absolutely agree (%)	Relatively agree (%)	Not sure (%)	Relatively disagree (%)	Absolutely disagree (%)
Q9	2.3	6.3	45.8	43.8	0.0
Q20	0.0	10.42	53.0	25.0	14.58
Q21	0.0	10.32	43.83	33.25	13.5
Q22	437	6.35	33.42	37.5	13.7
Q24	8.33	6.35	37.3	43.67	2.1

**Table 8:** Statistical situation of “Personal development” in motivation before the experiment.

Question items	Absolutely agree (%)	Relatively agree (%)	Not sure (%)	Relatively disagree (%)	Absolutely disagree (%)
Q11	14.38	10.42	24.00	41.44	8.43
Q12	0.00	10.42	31.25	54.17	4.17
Q17	2.04	2.04	22.92	64.67	6.45
Q18	0.00	4.47	34.50	50.40	8.43

**Table 9:** Statistical situation of “Intrinsic interest” in motivation after the experiment.

Question items	Absolutely agree (%)	Relatively agree (%)	Not sure (%)	Relatively disagree (%)	Absolutely disagree (%)
Q1	16.67	54.08	24.08	4.17	0.00
Q3	29.47	41.67	24.00	4.17	0.00
Q4	22.42	33.38	29.17	8.43	6.25
Q5	22.92	52.08	22.42	2.08	0.00
Q6	27.08	43.75	29.17	0.00	0.00
Q14	24.00	47.42	22.42	4.17	0.00
Q19	25.00	47.92	20.83	2.08	4.17

**Table 10:** Statistical situation of “Scores” in motivation after the experiment.

Question items	Absolutely agree (%)	Relatively agree (%)	Not sure (%)	Relatively disagree (%)	Absolutely disagree (%)
Q10	25.08	50.00	20.53	2.58	0.00
Q25	29.57	55.25	15.50	0.00	2.58
Q26	27.58	45.75	25.08	2.58	0.00
Q27	35.52	45.53	15.67	2.58	0.00

**Table 11:** Statistical situation of “Learning situation” in motivation after the experiment.

Question items	Absolutely agree (%)	Relatively agree (%)	Not sure (%)	Relatively disagree (%)	Absolutely disagree (%)
Q7	25.08	55.17	15.58	5.17	0.00
Q8	25.08	31.25	31.25	4.17	5.25

**Table 12:** Statistical situation of “Going abroad” in motivation after the experiment.

Question items	Absolutely agree (%)	Relatively agree (%)	Not sure (%)	Relatively disagree (%)	Absolutely disagree (%)
Q9	25.08	55.00	15.67	6.25	0.00
Q20	31.25	43.75	20.83	5.17	0.00
Q21	27.08	53.75	16.67	10.42	2.08
Q22	18.75	22.92	37.50	18.75	2.08
Q24	16.67	50.42	18.75	2.58	2.08

**Table 13:** Statistical situation of “Personal development” in motivation after the experiment.

Question items	Absolutely agree (%)	Relatively agree (%)	Not sure (%)	Relatively disagree (%)	Absolutely disagree (%)
Q11	37.55	50.00	12.55	0.00	0.00
Q12	41.57	39.58	10.42	4.17	4.17
Q17	41.57	37.50	18.55	2.58	0.00
Q18	35.52	45.83	14.58	4.17	0.00

**Table 14:** Pretest statistics of the experiment class and the control class.

	Class	*N*	Mean	Std. deviation	Std. error mean
Pretest scores	EC	48	11.43	2.836	0.409
	CC	50	11.17	2.869	0.406

**Table 15:** Independent sample test of pretest for the experiment class and the control class.

	Levene's test for equality of variances			t-test for equality of means				
Pretest scores		*F*	Sig.	*t*	Df	Sig. (2-tailed)	Mean difference	Std. error difference
	Equal variances assumed	0.014	0.092	0.412	97	0.681	0.236	0.576
	Equal variances not assumed			0.412	95.917	0.681	0.237	0.576

**Table 16:** Statistics of the experiment class and the control class.

	Class	*N*	Mean	Std. deviation	Std. error mean
Post-test scores	EC	48	13.64	2.702	0.390
	CC	50	11.17	3.062	0.433

## Data Availability

The labeled dataset used to support the findings of this study is available from the corresponding author upon request.
